# MiR-301a-3p Advances IRAK1-Mediated Differentiation of Th17 Cells to Promote the Progression of Systemic Lupus Erythematosus via Targeting PELI1

**DOI:** 10.1155/2021/2982924

**Published:** 2021-12-11

**Authors:** Shuaihantian Luo, Ruifang Wu, Qianwen Li, Guiying Zhang

**Affiliations:** Department of Dermatology, The Second Xiangya Hospital of Central South University, Changsha 410011, Hunan Province, China

## Abstract

Systemic lupus erythematosus (SLE) is a common autoimmune disease with high incidence in females. The pathogenesis of SLE is complex, and healing SLE has become a serious challenge for clinical treatment. Aberrant expression of miR-301a-3p involves the progressions of multiple diseases, and some studies have indicated that increased miR-301a-3p could induce the inflammatory injury of some organs. However, the role and molecular mechanism of miR-301a-3p in SLE remain unclear. In this study, the miR-301a-3p levels in peripheral blood mononuclear cells (PBMCs) of the patients with SLE and health subjects were measured with qRT-PCR. The ELISA assay was used to investigate the effect of miR-301a-3p on the levels of inflammatory factors in PBMCs, and flow cytometry assays were used to observe the effect of miR-301a-3p on the levels of CD4+ T cells and Th17 cells in PBMCs. Moreover, TargetScan, dual-luciferase reporter assay, and western blot were used to reveal the downstream targets and regulation mechanism of miR-301a-3p in SLE. The results showed that miR-301a-3p was significantly upregulated in PBMCs of the SLE patients, and increased miR-301a-3p could boost the expression of IL-6, IL-17, and INF-*γ* in PBMCs and promote the differentiation of Th17 cells. It was found that PELI1 was a target of miR-301a-3p, and PELI1 upregulation could effectively reverse the effect of miR-301a-3p on PBMCs. Besides, this study also found that miR-301a-3p could promote the expression of IRAK1 to involve the progression of SLE via targeting PELI1. In conclusion, this study suggests that increased miR-301a-3p serves as a pathogenic factor in SLE to promote IRAK1-mediated differentiation of Th17 cells via targeting PELI1.

## 1. Introduction

Systemic lupus erythematosus (SLE) is a common autoimmune disease which always involves the complications, such as the injury of skin, joints, and multiple organs [1, 2]. The incidence of SLE is increasing year by year. Statistically, the incidence of SLE in women is almost nine times than that in men [3]. The patients with SLE are characterized with diverse of immunologic abnormalities induced by the imbalance of T cell subset. Increased CD4+ T cells have also been confirmed as a marked event for SLE development [4]. Unfortunately, the symptoms SLE are complicated and recurrent, confounding attempts to determine the cause and develop effective methods for this disease. Moreover, limited new drug has been approved and applied in clinical treatment of SLE in recent years [5]. Thus, even with current therapeutic methods, the prognosis of the patients with SLE remains unsatisfactory.

MicroRNAs (miRNAs), the noncoding RNA, involve the translation of mRNA and thus play important roles in cellular vital movement [6]. Increasing studies have revealed that the dysfunctions of some miRNAs involve the development and deterioration of the autoimmune diseases [7, 8]. In recent years, several researches have indicated that miRNA profiling of the patients with SLE may exhibit obvious difference compared with that of the healthy persons. For instance, the study has indicated that miR-125b was significantly downregulated in the serums of the patients with SLE, and increased miR-125b could inhibit the autograph of peripheral blood mononuclear cells (PBMCs) to suppress the progression of SLE via directly targeting UVRAG [9].

Aberrant expression of miR-301a-3p is associated with multiple diseases ranging from cancer to inflammation. Increased miR-301a-3p can mediate the injury of organs induced by oxidative stress and inflammation [10]. However, the role of miR-301a-3p remains unclear. Thus, this study attempted to investigate the relationship of miR-301a-3p and SLE and reveal the molecular mechanism of miR-301a-3p in formation and development.

## 2. Materials and Methods

### 2.1. Pathological Samples

This study was approved by the ethics committee of the hospital. The PBMCs of the 15 patients with SLE and 15 health subjects were collected for next exploration.

### 2.2. Cell Culture and Transfection

30 mL of peripheral blood of the patients and healthy subjects was collected and then added with heparin anticoagulation (20 U/mL) for next experiments. Ficoll-Hypaque density gradient centrifugation (Solarbio, Beijing, China) was performed for PBMCs isolation. RPMI 1640 or DMEM was respectively used for cell culture of PBMCs and 293T, and 10% fatal bovine serum was used for maintaining cell growth. Besides, 100 g/mL penicillin G and streptomycin were also added into the medium to maintain cell growth. All cells were cultured in an incubator with 37°C and 5% CO_2_.

For cell transfection, when cellular confluence was at 70%, the 500 *μ*l serum-free medium containing 10 *μ*l Lipofectamine 2000 (Beijing Noble Ryder Technology Co., Ltd., Beijing, China) and 4 *μ*g of DNA or100 pmol RNA were added into each well. Finally, the cells were further cultured for 24 hours.

### 2.3. qRT-PCR

Total RNA of the cells was extracted with TRIzol reagent. The reverse transcription of RNA was performed with PrimeScript RT-PCR kit purchased from Beijing Zhijie Fangyuan Technology Co., Ltd., (Beijing, China). In brief, the preparation of reaction system was performed according to the instruction of the kit. After that, the qRT-PCR was performed according the following conditions: 95°C for 5 min, followed by 40 cycles of 95°C for 15 s, 62°C for 30 s, and 72°C for 30 s. Finally, the abundance of the RNA was calculated with 2^−(ΔΔCt)^ method. The primer sequences of the miR-301a-3p, PELI1, IRAK1, and U6 are listed in Table 1.

### 2.4. Western Blot

The cells were treated with RIPA lysis buffer and protease inhibitors on the ice for 30 min, and then the cells were collected with centrifugation (1000 r/min, 4°C for 10 min). Subsequently, the concentration of proteins in the supernatant was measured by BCA kit purchased from Shanghai Jining Biotechnology Co., Ltd. (Shanghai, China), and then it was boiled at 100°C for 5 min and added with loading buffer (5x). The proteins were separated with SDS-PAGE and then were translated on the PVDF membranes by wet translation methods. The membranes were blocked with 5% fat-free milk for 2 hours and then were incubated with the primary antibodies including anti-PELI1 (1 : 1000, Abcam, UK, ab199336), anti-IRAK1 (1 : 1000, Abcam, UK, ab208009), and *β*-actin (1 : 2000, Abcam, UK, ab8226) at 4°C overnight. After that, the membranes were washed with TBST for 3 times and then incubated with the second antibodies for 2 hours. Finally, the expression of the proteins was observed and quantified by a chemiluminescence detection system.

### 2.5. Flow Cytometry Assay

The proportion of Th17 cells in PBMCs was measured with flow cytometry assay. In brief, the PMBCs were incubated with anti-CD4 antibodies at 4°C for 30 min. Subsequently, the cells were fixed and permeabilized with Cytofix/Cytoperm at 4°C for 30 min and then washed with 0.05% saponin. After that, the cells were further incubated with anti-IL-17A for 1 hour. All options were performed in the dark.

### 2.6. Luciferase Reporter Assay

The downstream target of miR-301a-3p was searched with TargetScan and then was verified with luciferase reporter assay. In brief, the normal 3′-UTR sequence of PELI1 (PELI1-wt) and the related mutant sequence (PELI1-mut) were inserted into the luciferase vectors, respectively. Subsequently, the PELI1-wt or PELI1-mut was respectively cotransfected with miR-301a-3p inhibitors or related negative control with Lipofectamine 2000 (Thermo Fisher Scientific, MA, USA) into 293T cells. After incubation for 24 hours, the luciferase activity of miR-301a-3p on PELI1 was measured with Dual-Luciferase® Reporter Assay System (Promega Corporation).

### 2.7. ELISA Assay

ELISA assay was used to detect the levels of IL-17, IL-6, and IFN-*γ*. The assay was performed according the instruction of the ELISA kit (Shanghai Jining Biotechnology Co., Ltd., Shanghai, China), LD-96A microplate reader purchased from Shandong Leonard Intelligent Technology Co., Ltd., (Shandong, China) was used to detect the optical density (OD) values of the cells. The OD values of the cells were measured under 450 nm.

### 2.8. Statistical Analysis

The experiments in this study were preformed at least 3 times, independently. The data were analyzed by SPSS 20.0. Chi-squared test or ANOVA with Tukey's post hoc test was used to calculate the difference between the groups. *P* < 0.05 means that the statistical significance existed in two groups.

## 3. Results

### 3.1. MiR-301a-3p Was Significantly Upregulated in PBMC Cells of the Patients with SLE

To investigate the relationship of miR-301a-3p and SLE, the qRT-PCR was performed to evaluate the abundance of miR-301a-3p in PBMCs of the patients with SLE and health subjects. The study indicated that miR-301a-3p was obviously upregulated in the PBMCs of the patients (Figure 1, *P* < 0.01). This proof suggested that miR-301a-3p upregulation is related with the progression of SLE.

### 3.2. Downregulated MiR-301a-3p Inhibited the Expression of IL-6, INF-*γ,* and IL-17A in the PBMCs of the Patients

To observe the functions of miR-301a-3p on the progression of SLE, the miR-301a-3p inhibitors were transfected into PBMCs of the patients, and ELISA assay was performed to evaluate the expression levels of IL-6, INF-*γ,* and IL-17A. The results showed that the abundance of IL-6, INF-*γ,* and IL-17A increased significantly in PBMCs transfected with miR-301a-3p inhibitors (Figure 2, *P* < 0.01). Those proofs suggest that increased miR-301a-3p involves in the progression of SLE.

### 3.3. PELI1 Was a Downstream Target of MiR-301a-3p

To delve the regulation mechanism of miR-301a-3p in the development of SLE, the downstream factors of miR-301a-3p were searched with online database, such as TargetScan. The results showed that PELI1 was a potential target of miR-301a-3p. Moreover, the results of dual-luciferase reporter assay showed that miR-301a-3p could obviously decrease the luciferase activity of the cells transfected with PELI1-wt vectors, while having little effect on the luciferase activity of 293T cells transfected with PELI1-mut vectors (Figure 3(a), *P* < 0.01). Moreover, it was also found that PELI1 was downregulated in the PBMCs of the patients with SLE (Figure 3(b), *P* < 0.01).

### 3.4. Downregulated PELI1 Reversed the Effect of MiR-301a-3p Silence on the PBMCs of the Patients

To further confirm whether PELI1 involves the regulation of miR-301a-3p on SLE, the inhibitors of miR-301a-3p and si-PELI1 were cotransfected into the PBMCs of the patients, and the change of the inflammatory factors in the PBMCs of the patients was observed by ELISA. The results showed that the levels of IL-6, INF-*γ,* and IL-17A were partly reversed in the cells cotransfected with the inhibitors of miR-301a-3p and si-PELI1 compared with the cells transfected with miR-301a-3p inhibitors (Figures 4(a)–4(c), *P* < 0.01). Moreover, it was also found that the proportion of Th17 cells in the PBMCs of the patients transfected with miR-301a-3p inhibitors significantly decreased, while PELI1 silence could partly reverse those phenomena (Figure 4(d), *P* < 0.01).

### 3.5. MiR-301a-3p Promoted the Progression of SLE via Targeting PELI1

To further illustrate the molecular mechanism of miR-301a-3p in SLE, the miR-301a-3p inhibitors and si-PELI1 vectors were cotransfected into the S-PMSCs, and the expression of IRAK1 and activity of NF-*κ*B pathway were observed by western blot. The results showed that miR-301a-3p downregulation obviously inhibited the expressions of IRAK1, p-IRAK1, and p-P65 (Figure 5, *P* < 0.01). However, PELI1 silence could partly reverse the effect of decreased miR-301a-3p on the expression of IRAK1, p-IRAK1, and p-P65. Those observations suggested that miR-301a-3p could directly target PELI1 to promote the IRAK1-induced activation of NF-*κ*B pathway.

## 4. Discussion

SLE is a serious autoimmune disease which threatens the health of females, and there are few perfect strategies for SLE healing [11]. MiR-301a-3p plays an important role in inducing multiple inflammatory injury, while its role in SLE remains unclear [12]. This study investigated the abundance of miR-301a-3p in PBMCs and revealed the role of miR-301a-3p in the progression of SLE. Moreover, the pathogenic mechanism of miR-301a-3p was illustrated by exploring the downstream regulatory pathway.

MiRNA dysfunction has been contributed as an important reason leading the progression of inflammation and stress injury [13, 14]. In this study, it was found that miR-301a-3p was obviously upregulated in PBMCs of the patients with SLE. MiR-301a-3p serves as an inflammatory factor to mediate the injury of tissues, and aberrant expression of miR-301-3p may be associated with the formation and development of autoimmune diseases [15]. The research showed that increased miR-301a-3p can induce the kidney injury via promoting cell apoptosis [16]. This study confirmed that downregulated miR-301a-3p could inhibit the expressions of IL-6, INF-*γ,* and IL-17A. Therefore, this study suggested that miR-301a-3p upregulation is related with the progression of SLE.

MiRNA is characterized with translation repression of some proteins via targeting the 3′-UTR of the related mRNAs [17]. MiR-301a can also directly bind with Runx3 to promote the malignant progression of lung cancer [18]. According to the TargetScan and luciferase assay, PELI1 was identified as a downstream target of miR-301a-3p, and downregulated PELI1 was also found in PBMCs, suggesting that PEL11 takes part in the pathogenic pathways of miR-301a-3p on SLE. PELI1 is an E3 ubiquitin ligase enzyme which can regulate the maturation and differentiation of T cells via mediating protein ubiquitin [19]. The study has indicated that PELI1 serves as a negative regulator to block the deterioration of SLE [20]. Hence, this study suggests that miR-301a-3p could drive the progression of SLE via targeting PELI1.

Th17 is one of the subsets of effector CD4+ T cells, which is associated with the formation and deterioration of chronic inflammatory diseases [6]. Aberrant Th17 level has been proved as the major reason for SLE progression. In this study, it was found that miR-301-3p could promote the differentiation of Th17 cells. Several studies have indicated that IL-17 is significantly upregulated in the serum of the patients with autoimmune disease, and upregulated IL-17 plays an autoantibody role in triggering the progression of SLE. This study also confirmed that the miR-301-3p promoted the expression of IL-17 in PBMCs. He et al. have indicated that miR-301a could boost the expression of IL-17A and TNF-*α* to induce the inflammation of intestinal mucosa [21]. Thus, those proofs suggest the miR-301a-3p upregulation enhances the SLE via driving the differentiation of Th17 and promoting the expression of IL-17.

Although miR-301a-3p cells have been verified to involve the differentiation of Th17 cells via targeting SNIP1, this study also found a new regulation mechanism of miR-301a-3p on the differentiation of Th17 in the progression of SLE [12]. The study has indicated that PELI1 could induce the K-63 ubiquitination of IRAK1 to impede the progression of IRAK1 [9]. In this study, it was found that miR-301a-3p downregulation could effectively inhibit the expression of IRAK1, and PELI1 silence could partly reverse this phenomenon. IRAK1 serves as an attractant for development of SLE, and aberrant expression of IRAK1 also promoted the imbalance of the expression level of Th17, and thus has been thought as a biomarker for SLE [22]. Recently, several studies have indicated that abnormal activation of NF-*κ*B pathway may be related to upregulated IRAK4. Meng et al. have found that IRAK4 is extremely upregulated in nasopharyngeal carcinoma cells, and S100A14 could inhibit NF-*κ*B pathway to impede the progression of the cancer via targeting IRAK4 [23]. In this study, it was found that miR-301a-3p silence could effectively inactivate the NF-*κ*B pathway, and this phenomenon could be reversed by decreased PELI1. Activated NF-*κ*B pathway is associated with the progression of some inflammations and stress injuries, and thus it has been thought as a promising target for drug development. For SLE, NF-*κ*B pathway also plays a key role in its formation and development [24]. The study has showed that miR-146a upregulation could effectively improve the kidney injury of the mice via inhibiting NF-*κ*B pathway [25]. Therefore, this study supports that miR-301a-3p could activate the IRAK1-mediated NF-*κ*B pathway to promote the progression of SLE via targeting and downregulating PELI1.

## Figures and Tables

**Figure 1:** MiR-301a-3p was significantly upregulated in the PBMCs of the patients with SLE (^*∗∗*^*P* < 0.05).

**Figure 2:** MiR-301a-3p silence inhibited the expressions of IL-6, IL-17, and INF-*γ*. (a–c) The relative expression levels of IL-6, IL-17, and INF-*γ* were measured with ELISA assay (^*∗∗*^*P* < 0.05).

**Figure 3:** PELI1 was a target of miR-301a-3p and was significantly downregulated in PBMCs of the patients with SLE. (a) The binding effect of miR-301a-3p and PELI1 was observed by luciferase assay. (b) The mRNA level of PELI1 in PBMCs of the patients with SLE was measured by qRT-PCR (^*∗∗*^*P* < 0.05).

**Figure 4:** PELI1 silence partly reversed the effect of inhibited miR-301a-3p on the levels of inflammatory factors in the PBMCs of the patients and the differentiation of Th17 cells. (a–c) The relative expression levels of IL-6, IL-17, and INF-*γ* were measured with ELISA assay. (d) The proportion of Th17 in the PBMCs of the patients was evaluated by flow cytometry assay (^*∗∗*^*P* < 0.05).

**Figure 5:** MiR-301a-3p directly targeted PELI1 to promote the IRAK1-induced activation of NF-*κ*B pathway. (a) The relative expression level of miR-301a-3p was measured by qRT-PCR. (b–f) The relative expression levels of PELI1, IRAK1, p-IRAK1, and p-P65 were measured by western blot (^*∗∗*^*P* < 0.05).

**Table 1:** Primer sequence.

Name of primer	Sequence
MiR-301a-3p-F	5′-ATGATGGGGTGGTATTTGTTTAG-3′
MiR-301a-3p-R	5′- TCCTTCAAACTTAGAAATGTCAAG-3′
PELI1-F	5′-TGTAGTAACTGACACGGTTCCT-3′
PELI1-R	5′-TCCATCTGATGTCTTCCATTTGG-3′
IRAK1-F	5′-ATGTCGTCCTGGGATATCGGA-3′
IRAK1-R	5′-TTAGTTGTGAGCGTTGGTCT-3′
U6-F	5′-CTCGCTTCGGCAGCACA-3′
U6-R	5′-AACGCTTCACGAATTTGCGT-3′

## Data Availability

The data that supported the findings of this study are available on reasonable request from the corresponding author.
